The article "Ginkgolide B inhibits lung cancer cells promotion via beclin-1-dependent autophagy" was retracted in 2023. Reasons: duplicated images; overlap with earlier publications; unreliable data; concerns about the images.

# Ginkgolide B inhibits lung cancer cells promotion via beclin-1-dependent autophagy

**DOI:** 10.1186/s12906-020-02980-x

**Published:** 2020-06-23

**Authors:** Xuan Wang, Qi-Hui Shao, Hao Zhou, Jun-Lu Wu, Wen-Qiang Quan, Ping Ji, Yi-Wen Yao, Dong Li, Zu-Jun Sun

**Affiliations:** 1 Department of Pharmacy, Putuo People’s Hospital, Shanghai, 200060 China; 2 Department of Traditional Chinese Medicine, Shanghai Tongji Hospital, Tongji University School of Medicine, Shanghai, 200065 China; 3 Department of Clinical Laboratory, Shanghai Tongji Hospital, Tongji University School of Medicine, Shanghai, 200065 China

**Keywords:** *Ginkgolide B*, Light chain 3B, NLRP3, Beclin-1, Autophagy

## Abstract

**Background:**

*Ginkgolide B* (GKB) is a major active component of the extracts of *Ginkgo biloba* leaves, and it has been used as an anti-cancer agent. However, it is unknown whether GKB has the therapeutic effects on lung cancer. Here, we studied the effects of GKB on lung cancer cells.

**Methods:**

The effects of GKB on lung cancer cell proliferation and invasion were analyzed by cell counting kit (CCK-8) and cell invasion assays, respectively. Apoptosis was detected by flow cytometry. Western blot analysis was used to confirm the expression of autophagy-associated proteins in GKB-treated cells. Immunofluorescence analysis was used to analyze the level of light chain 3B (LC3B).

**Results:**

Treatment with GKB time-dependently inhibited the proliferation and decreased the invasive capacity of A549 and H1975 cells. GKB induced apoptosis of these cells, but there was no significant effect on apoptosis compared to the control treatment. GKB-induced inhibition of cell proliferation and GKB-induced cell death were due to autophagy rather than apoptosis. GKB-induced autophagy of lung cancer cells was dependent on beclin-1, and autophagy-induced inhibition of the NLRP3 inflammasome contributed to the anti-tumor effect of GKB.

**Conclusions:**

GKB-mediated autophagy of lung cancer cells is beclin-1-dependent and results in inhibition of the NLRP3 inflammasome. Therefore, GKB might be a potential therapeutic candidate for the treatment of lung cancer.

## Background

Lung cancer is the most common type of malignant tumor and the leading cause of cancer-related death worldwide [1]. Currently, the majority of lung cancer patients are diagnosed when they have advanced stage of the disease and have therefore missed the opportunity to undergo surgery to treat the cancer [2]. Chemotherapy is the main treatment for patients with advanced lung cancer. However, the efficacy of chemotherapy for lung cancer is limited, and drug resistance is common. Therefore, developing and discovering new agents to treat lung cancer is urgent.

The article "Ginkgolide B inhibits lung cancer cells promotion via beclin-1-dependent autophagy" was retracted in 2023. Reasons: duplicated images; overlap with earlier publications; unreliable data; concerns about the images.

In recent years, anti-cancer agents extracted from traditional Chinese herbal medicines have attracted much attention. *Ginkgolide B* (GKB), the major active component of the extracts *of Ginkgo biloba* leaves, has been used in Chinese herbal medicine for centuries. It has been shown to exert a wide range of biological activities, including anti-oxidant and anti-lipoperoxidative properties, which are considered to play an important role in the prevention of cancer [3]. It was reported that GKB could inhibit the proliferation of human breast cancer cells via its effect on the peripheral-type benzodiazepine pathway, which plays an important role in steroid hormone regulation. GKB has significant anti-proliferative and cytotoxic effects on human hepatocellular carcinoma cells [4, 5]. In vivo experiments have suggested that GKB can promote apoptosis by activating caspase-3 in cancer cells in the oral cavity rats, indicating that it has pro-apoptotic effects for this type of cancer [6]. GKB has also been shown to prevent benzo [a) pyrene-induced forestomach carcinogenesis in mice [7]. Previous studies showed that GKB inhibits bladder and ovarian cancer [8, 9]. However, although multiple biological functions of GKB have been identified, little is known about the effects of GKB on lung cancer cells.

Autophagy is a means of cell suicide that is characterized by the isolation of cytoplasmic material in vacuoles for bulk degradation by lysosomal enzymes [10]. It has been reported that autophagy can be induced by a variety of stimuli, such as ionizing radiation, endoplasmic reticulumstress, and chemotherapeutic drugs [10]. Previous studies have indicated that members of the B-cell lymphoma (Bcl)-2 family can regulate multiple intracellular pathways and they have a strong impact on autophagy, which may due to their interaction with the autophagy regulator beclin-1 [11–15]. In prostate cancer cells with high Bcl-2 expression, > 60% of cells die by autophagy, which can be blocked by the autophagy inhibitor 3-methyladenine (MA) or small interfering RNA (siRNA) targeting beclin-1 (the mammalian homolog of yeast Atg6) or Atg5 [16]. Lack of autophagy-related proteins can lead to mitochondrial dysfunction and DNA release into the cytoplasm, this promotes the activation of the NLR family pyrin domain-containing 3 (NLRP3) inflammasome [17], which is the most extensively studied inflammasome. As a potentially important chemotherapeutic drug, the effects of GKB on the autophagy of lung cancer cells and the precise molecular mechanisms underlying these effects are unknown.

In this study, we investigated the role of GKB chemotherapy in lung cancer cell lines and explored the precise molecular mechanisms. Our results demonstrated that GKB can inhibit the proliferation and invasion of lung cancer cells in vitro and induce beclin-1-dependent autophagy. These effects might due to autophagy-induced inhibition of the NLRP3-related inflammasome.

The article "Ginkgolide B inhibits lung cancer cells promotion via beclin-1-dependent autophagy" was retracted in 2023. Reasons: duplicated images; overlap with earlier publications; unreliable data; concerns about the images.

## Material and methods

### Cell culture and reagents

Lung carcinoma cell lines H1975 and A549 were purchased from the American Type Culture Collection and cultured in Dulbeccos’s modified Eagle’s medium (DMEM) (Hyclone Laboratories, Inc., South, UT, USA) supplemented with 10% fetal bovine serum (FBS) (Invitrogen, Grand Island, NY, USA), 100 U/mL penicillin and 100 U/mL streptomycin (Hyclone Laboratories, Inc., South, UT, USA), and maintained in a humidified 5% CO_2_ atmosphere at 37 °C. GKB (CAS No.15291–76-6, BN52022) was obtained from the Tauto Biotech Co., Ltd., Shanghai, China, and dissolved in dimethyl sulfoxide (DMSO), chloroquine (S4157, Selleck, Houston, USA), 3-Methyladenine (S2767, Selleck, Houston, USA), GFP-LC3B virus vector (Genomeditech, Shanghai, China).

### Cell proliferation and apoptosis assay

A cell proliferation assay was performed using the cell counting kit (CCK)-8 (DojinDo, Tokyo, Japan) with both A549 and H1975 cells. In brief, 1000 cells were seeded into a 96-well plate and treated with 200 mg/L GKB or DMSO for 0, 24, 48, and 72 h. Absorbance at 450 nm was measured using a microplate reader (ThermoFisher Scientific, Waltham, MA, USA). Apoptotic cells were assessed as previously described [18].

### Cell invasion assay

Cell invasion assays were performed as previously described [19]. A549 and H1975 cells were suspended in serum-free DMEM and then 0.1 mL of these solutions were added to the inserts. Next, 0.7 mL serum-containing medium with or without GKB (200 mg/L) was added to the lower chambers. The chemoattractant used was 10% fetal calf serum. The chambers were then assembled and incubated for 24 h at 37 °C. Thereafter, non-invading cells were scrubbed off the upper surface of the membrane. The invaded cells on the lower surface were fixed with 100% methanol, stained with 0.1% crystal violet solution (Sigma-Aldrich, St. Louis, MO, USA), and counted using a microscope (based on five random fields). The relative migration was calculated based on the ratio of the number of invaded cells in the GKB group versus the number of invaded cells in the DMSO control group.

### Colony formation assay

A549 and H1975 cells were plated at a low density (5 × 10^2^ cells per well) in 6-well plates. They were treated with 50, 100, or 200 mg/L GKB or DMSO. They were then incubated for 14 days at 37 °C and 5% CO_2_ in a humidified atmosphere. The colonies were then fixed with 2% paraformaldehyde, stained with a 0.05% crystal violet solution (Sigma-Aldrich, St. Louis, MO), and counted using an inverted microscope.

The article "Ginkgolide B inhibits lung cancer cells promotion via beclin-1-dependent autophagy" was retracted in 2023. Reasons: duplicated images; overlap with earlier publications; unreliable data; concerns about the images.

### Western blot analysis

Western blot was assessed as previously described [18]. The following primary antibodies (Cell Signaling Technology) were used: rabbit anti-proliferating cell nuclear antigen (PCNA (#13110), rabbit anti-caspase3 (#9664), rabbit anti-LC3B (#3868), rabbit anti-beclin-1 (#3495), and rabbit anti-Bcl-2 (#2872). HRP-conjugated goat anti-rabbit (Santa Cruz) or rabbit anti-mouse (Dako, Carpinteria, CA, USA) was used as secondary antibody. After washing the membranes using TBS with Tween 20 (TBS-T), the immunereactive bands were visualized using a chemiluminescence substrate.

### Immunofluorescence assay

Immunofluorescence was assessed as previously described [18]. The monoclonal mouse anti-LC3B (Santa Cruz Biotechnology, Inc., Santa Cruz, CA, USA) antibody was overnight. PE-labeled (1:100) anti-rabbit IgG served as the secondary antibody. The slides were evaluated (based on five random fields) with fluorescence microscope Nikon Eclipse Ti-S fluorescence microscope (Nikon, Tokyo, Japan).

### Effects of beclin-1 specific siRNA

Expression of beclin-1 in the cell lines was temporarily silenced using small interfering RNA (siRNA) of beclin-1. The sense and antisense strands of beclin-1 siRNA were: 5-CCCAGGAGGAAGAACUAATT-3 and 5-UUAGUCUCU UCCUCCUGGGTC-3. Briefly, 2 × 10^5^ tumor cells were seeded in the wells of six-well plates and cultured in DMEM. The next day, the cells were transfected with human siRNA (HIPPOBIO. Co., Huzhou, China) at different concentrations according to the manufacturer’s instructions. The negative control consisted of siRNA with no homology to known sequences from humans. Cells were incubated in complete DMEM medium at 37 °C in an atmosphere of 5% CO_2_. Western blot was used to test beclin-1 expression and further experiments were carried out.

### Enzyme-linked immunosorbent assay (ELISA)

To elucidate whether GKB inhibits lung cancer cells by inhibiting autophagy in order to inhibit NLRP3 inflammasome activation, we treated H1975 cells with the autophagy inhibitor 3-MA. Lipopolysaccharide (LPS) was used to activate the NLRP3 inflammasome. Next, GKB or DMSO was added to the cells for 24 h. The levels of interleukin-1 (IL-1β) and interleukin-8 (IL-18) were measured using ELISA kits (CUSABIO, Wuhan, China) according to the instructions provided by the manufacturer.

### Statistical analysis

The data were obtained from at least three independent experiments and presented as the mean ± SEM. Differences in means were analyzed using Student’s t-test and one-way analysis of variance. *P* < 0.05 denoted statistical significance. All statistical analyses were performed with SPSS22 statistical software (SPSS Inc., Chicago, IL, USA).

The article "Ginkgolide B inhibits lung cancer cells promotion via beclin-1-dependent autophagy" was retracted in 2023. Reasons: duplicated images; overlap with earlier publications; unreliable data; concerns about the images.

## Results

### GKB inhibits the proliferation and invasion of lung cancer cells in vitro but does not promote apoptosis

Previous studies have shown that GKB inhibits bladder and ovarian cancer [8, 9]. To assess whether the GKB-induced anti-tumor effect is relevant in lung cancer cells, we treated H1975 and A549 cells with GKB. GKB time-dependently inhibited the proliferation (Fig. 2a). To determine the effects of GKB on the cell invasion and colony-formation abilities of lung tumor cells, H1975 and A549 cells were grown on Matrigel and in 6-well plates, respectively. After 24 h, GKB significantly decreased the invasive capacity (Fig. 2b) as well as dose-dependently inhibiting the ability to form colonies of A549 and H1975 cells after 14 days (Fig. 2c).

To better understand the mechanism underlying the anti-tumor effect of GKB, we first examined apoptosis by flow cytometry. Upon GKB treatment, H1975 and A549 cells exhibited an increased percentage of apoptotic cells, but no significant difference was detected when compared to the control (Fig. 2d). This suggests that apoptosis may not be the major mechanism underlying the anti-tumor effect of GKB.

### GKB induces autophagy but not apoptosis in lung tumor cells

Autophagy is an important mechanism of cell self-destruction and has a crucial role in tumorigenesis processes [10]. To assess whether the anti-tumor effect of GKB treatment is due to the induction of autophagy, we analyzed the expression of proteins known to be involved in cell autophagy. The expression of beclin-1, p62, and LC3B proteins was strongly induced in response to 200 mg/L GKB treatment in lung tumor cells in a time-dependent manner by western blot analysis (Fig. 3a). This result was confirmed by immunofluorescence analysis of LC3B, which significantly increased in the cells after GKB treatment (Fig. 3b). In addition, the expression of PCNA and Bcl-2 decreased in a time-dependent manner in GKB-treated A549 and H1975 cells (Fig. 3a).

To elucidate the role of autophagy in the GKB-induced inhibition of invasion and colony formation of lung cancer cells, we pretreated H1975 cells with3-MA, a selective autophagy inhibitor. Autophagy inhibition significantly interfered with the GKB-induced decrease in the number of invasive cells in vitro (Fig. 4a), as well as interfering with the GKB-induced decreased in the number of cell colonies (Fig. 4b). The expression of beclin-1, p62, and LC3B proteins was also strongly interfered with by 3-MA pretreatment of lung tumor cells based on the western blot analysis (Fig. 5a). A similar result was obtained based on the immunofluorescence analysis of LC3B (Fig. 5b).

The article "Ginkgolide B inhibits lung cancer cells promotion via beclin-1-dependent autophagy" was retracted in 2023. Reasons: duplicated images; overlap with earlier publications; unreliable data; concerns about the images.

### GKB induces beclin-1-dependent autophagy in lung cancer cells

It has been reported that beclin-1 is increased in some cells and plays a pivotal role in inducing cell autophagy. The western blot analysis showed that beclin-1 expression in GKB-treated lung cancer cells was significantly regulated, which was reversed by 3-MA pretreatment (Fig. 5a, b). Next, we wanted to know whether beclin-1 is involved in GKB-induced cell autophagy. To this end, we transfected H1975 cells with siRNA targeting beclin-1 (a western blot analysis confirmed the reduction of beclin-1) (Fig. 6a). GKB-induced autophagy was decreased in these cells compared to the control cells, indicating that beclin-1 is required for the signal transduction underlying GKB-induced cell autophagy (Fig. 6b).

### Autophagy-induced inhibition of the NLRP3 inflammasome contributes to the anti-tumor effect of GKB

The NLRP3 inflammasome plays a central role in tumorigenesis and development [20]. To investigate the mechanism of the anti-tumor effect of GKB, we examined NLRP3 inflammasome activation in lung cancer cells. Treatment of H1975 cells with GKB for 24 h significantly reduced NLRP3 expression (Fig. 7a). Previous research showed that autophagy mediates inhibition of NLRP3 inflammasome activation [21]. To elucidate whether or not the inhibition effect of GKB on NLRP3-related inflammasome activation (which leads to pro- IL-1β and pro-IL-18 being cleaved to creat mature bioactive forms) depends on autophagy modulation, we treated lung cancer cells with an autophagy inhibitor. Lipopolysaccharide (LPS), which primes the expression of NLRP3, IL-1β, and IL-18 was used as an NLRP3-related inflammasome activator. The levels of both IL-1β and IL-18 in the H1975 cells were obviously elevated after stimulation with LPS, according to the enzyme-linked immunosorbent assay (ELISA) results (Fig. 7b). As expected, the GKB-induced inhibition of IL-1β and IL-18 expression were reversed by the autophagy inhibitor 3-MA according to the ELISA results. In order to determine whether beclin 1 knock-down is having any effect on autophagy-induced inhibition of NLRP3 inflammasome, western blot and ELISA were used to determine the level of NLRP3, IL-1β, and IL-18 proteins. These results showed that GKB-induced inhibition of NLRP3 inflammasome can be reversed by beclin-1 knockdown in H1975 cells (Fig. 7c, d).

## Discussion

GKB is a major active component of the extracts of *Ginkgo biloba* leaves, and it can also be synthesized chemically as a monomer, which exhibits the same activities (Fig. 1a, b, c). In this study, we investigated the effects of GKB in lung cancer cells in vitro. Our results showed that GKB can inhibit the proliferation and invasion of lung cancer cells*.* GKB induced autophagy, but not apoptosis, of lung cancer cells, which was dependent on beclin-1. This may contribute to the anti-tumor effect of GKB in a process involving autophagy-induced inhibition of the NLRP3 inflammasome.

The article "Ginkgolide B inhibits lung cancer cells promotion via beclin-1-dependent autophagy" was retracted in 2023. Reasons: duplicated images; overlap with earlier publications; unreliable data; concerns about the images.

**Fig. 1:** Structure and features of *ginkgolide B* (GKB). **a** Chemical structure of GKB. **b** GKB 3D conformations (visualized by Jmol; http://www.jmol.org) generated in the 3D mol2 format. **c** Drug-like properties

Previous studies showed that GKB inhibits bladder and ovarian cancer [8, 9]. We found that GKB can time-dependently inhibit the proliferation of A549 and H1975 cells (Fig. 2a). We also found that the expression of PCNA, a cellular marker of proliferation, and Bcl-2, a cellular anti-apoptosis marker, decreased in a time-dependent manner in GKB-treated A549 and H1975 cells (Fig. 3a). The results of the cell invasion and colony-formation assays showed that GKB significantly and dose-dependently decreased the invasive capacity and colony-formation ability (Fig. 2b, c). Thus, GKB decreases the proliferation, invasion, and colony formation of lung cancer cells, which constitutes strong evidence that GKB acts as a tumor inhibitor. Although the percentage of apoptotic cells among the A549 and H1975 cells increased after GKB treatment, there was no significant difference compared to the control group (Fig. 2d), which suggests that promoting apoptosis may not be the major mechanism underlying anti-lung cancer effect of GKB. Apoptosis and autophagy are well-characterized processes that contribute to the maintenance of cellular and tissue homeostasis. The crosstalk between apoptosis and autophagy has been documented in various physiological and pathological conditions [22, 23]. To assess whether the anti-tumor effect of GKB treatment is due to the induction of autophagy, we analyzed the expression of proteins known to be involved in cell autophagy. We found that the expression of LC3B protein was strongly and time-dependently upregulated after treatment with GKB in lung tumor cells, as beclin-1 and p62 proteins levels were (Fig. 3a). This result was further confirmed by immunofluorescence analysis (Fig. 3b). Furthermore, autophagy inhibition significantly interfered with the GKB-induced decrease in the number of invasive cells in vitro (Fig. 4a) and the decrease in the number of cell colonies (Fig. 4b). However, the changes in the expression of the above proteins were reversed by 3-MA (Fig. 5a, b). From these results, we can conclude that autophagy may play a critical role in GKB-induced inhibition of lung cancer in vitro.

The article "Ginkgolide B inhibits lung cancer cells promotion via beclin-1-dependent autophagy" was retracted in 2023. Reasons: duplicated images; overlap with earlier publications; unreliable data; concerns about the images.

**Fig. 2:** *Ginkgolide B* (GKB) inhibited the proliferation, invasion and colony formation of lung cancer cells in vitro and induced apoptosis*.***a** GKB significantly inhibited the proliferation of lung cancer cells. **b** GKB significantly inhibited the invasion of lung cancer cell. **c** GKB significantly inhibited the colony formation of lung cancer cells. Scale bar, = 200 μm. **d** Cancer cells were incubated with GKB for 48 h, and then apoptotic cells (stained with annexin V and propidium iodide) were detected by flow cytometry. Results are presented as mean ± SEM of three independent experiments. *P < 0.05, **P < 0.01, ***P < 0.001, compared to the dimethyl sulfoxide (DMSO) only group

**Fig. 3:** Anti-tumor effect of *ginkgolide B* (GKB) is due to the induction of autophagy. **a** Western blot analysis of the expression of Bcl-2, PCNA, beclin-1, p62, LC3B, and β-actin in H1975, and A549 cells after stimulation with GKB for the indicated time periods. **b** Immunofluorescence staining showing the subcellular localization and expression of LC3B in H1975 and A549 cells. Scale bar, = 20 μm

**Fig. 4:** Role of autophagy in GKB induced inhibition of invasion and colony formation of lung cancer cells. **a** Cell invasion analysis to assess the role of autophagy in GKB induced inhibition invasion of H1975 cells. **b** Colony formation analysis to assess the role of autophagy in GKB induced inhibition of the proliferation of H1975 cells. Data shown represent the mean ± SEM of three independent experiments. *P < 0.05, compared to the dimethyl sulfoxide (DMSO) only group

**Fig. 5:** Signaling pathways underlying *Ginkgolide B* (GKB) induced autophagy of lung cancer cells. **a** Western blot analysis of the proteins expression in lung cancer cells pretreated with 3-MA. **b** Immunofluorescence analysis of the expression of the LC3B protein in lung cancer cells pretreated with 3-MA

Beclin-1 (the mammalian ortholog of yeast Atg6) has an evolutionarily conserved role in macroautophagy [24]. Emerging lines of evidence suggest that beclin-1 is a novel substrate of caspases [25]. To assess the role of beclin-1 in GKB-induced autophagy, we examined the expression levels of p62 and LC3B (which is involved in autophagy) in beclin-1 knockdown lung cancer cells and found that p62 and LC3B (GKB-induced autophagy) were decreased in the beclin-1 knockdown group compared to the control group (Fig. 6b). From these results, we can conclude that beclin-1 is required for the signal transduction underlying GKB-induced cell autophagy.

The article "Ginkgolide B inhibits lung cancer cells promotion via beclin-1-dependent autophagy" was retracted in 2023. Reasons: duplicated images; overlap with earlier publications; unreliable data; concerns about the images.

**Fig. 6:** *Ginkgolide B* (GKB) induced autophagy that is dependent on beclin-1 in lung cancer cells. **a** Western blot analysis of the efficiency of beclin-1 knockdown. **b** Western blot analysis of the proteins expression in beclin-1-knockdown lung cancer cells

The NLRP3 inflammasome is the most extensively studied inflammasome. NLRP3 is triggered by a variety of stimuli, including infection, tissue damage, and metabolic dysregulation, and then activated through an integrated cellular signaling pathway. To form the inflammasome, NLRP3 combines with ASC and pro-caspase-1, which triggers proteolytic processing of pro-caspase-1 into its active form, caspase-1. Caspase-1 subsequently cleaves pro-IL-1β and pro-IL-18 to create the mature bioactive forms [26]. The ASC-mediated inflammation signaling pathway has been shown to be associated with tumorigenesis [27]. Wang et al. reported that IL-18 and IL-1β secretion was elevated due to NLRP3 inflammasome activation in A549 lung adenocarcinoma cells, and they suggested that a combination of IL-18 and IL-1β may have therapeutic potential [28]. In vivo research indicated that nanoparticles such as silica and asbestos can result in the overexpression of NLRP3 inflammasomes, and the secretion of caspase-1 and IL-1β in an animal model of lung cancer [29]. Autophagy has been shown to play a number of roles in regulating inflammasome activation, from the removal of inflammasome-activating endogenous signals to the sequestration and degradation of inflammasome components [30, 31]. Dysfunction of autophagy plays a role in determining the fate of inflammasome related IL-1β, which is concentrated in autophagosomes [32, 33]. Studies have shown that loss or impairment of autophagy in macrophages and dendritic cells can lead to hypersecretion of IL-1α, IL-1β and IL-18 [34]. Many regulatory mechanisms have been identified to attenuate NLRP3 inflammasome signaling at multiple points in the signaling pathway. Among them, the induction of selective mitochondrial autophagy, which results in selective clearance of damaged mitochondria in cells, can negatively regulate NLRP3 inflammasome activation [35, 36]. In the present study, we found that treatment of H1975 cells with GKB significantly reduced NLRP3 expression (Fig. 7a). In addition, GKB significantly inhibited IL-1β and IL-18 secretion by the H1975 cells (Fig. 7b). To elucidate whether or not the inhibition of NLRP3 inflammasome activation by GKB depends on autophagy modulation, we treated the lung cancer cells with an autophagy inhibitor (3-MA) and knocked down beclin-1. As expected, GKB-induced inhibition of NLRP3, IL-1β, and IL-18 expression was reversed by the autophagy inhibitors 3-MA or beclin-1 knock-down (Fig. 7b, d). These findings suggest that beclin-1-dependent autophagy is responsible for GKB-mediated inhibition of the NLRP3 inflammasome.

The article "Ginkgolide B inhibits lung cancer cells promotion via beclin-1-dependent autophagy" was retracted in 2023. Reasons: duplicated images; overlap with earlier publications; unreliable data; concerns about the images.

**Fig. 7:** Autophagy-induced inhibition of the NLRP3 inflammasome contributes to the anti-tumor effect of *Ginkgolide B* (GKB). **a** Western blot analysis of the expression of NLRP3 protein in H1975 cells treated with GKB for 24 h. **b** ELISA analysis of the expression of IL-1β and IL-18 protein after LPS was used as an NLRP3 inflammasome activator in H1975 cells. **c** Western blot analysis of the expression of NLRP3 protein in beclin-1 knock-down H1975 cells. **d** ELISA analysis the expression of IL-1β and IL-18 protein in beclin-1-knockdown H1975 cells. Data shown represent the mean ± SEM of three independent experiments. ***P < 0.001, compared to the dimethyl sulfoxide (DMSO) only group

There are several limitations in this study. The anti-apoptotic subfamily includes Bcl-2, Bcl-extra large (XL), Bcl-W, myeloid cell leukemia1 (Mcl-1), and Burkholderia lethal factor 1 (BLF1)/A-1 [15, 37–40], but whether these other proteins are involved in GKB-induced lung cancer cell autophagy remains to be studied. Besides the beclin-1 pathway, other mechanisms or pathways may also be involved in GKB-induced autophagy. In the future, we plan to elucidate the other precise mechanisms underlying the regulation of autophagy by GKB. Lastly, due to the poor water-solubility of GKB, it is difficult to verify its effect on of autophagy in lung cancer in vivo.

## Conclusions

Taken together, our results showed that GKB acted as an anti-tumor agent to suppress the proliferation, invasion, and colony formation of lung cancer cells. GKB can induce autophagy, but not apoptosis, in lung tumor cells, which depends on beclin-1. The anti-tumor effect of GKB may be related to the inhibition of NLRP3-related inflammation (Fig. 8). Our finding suggested that GKB is a potential therapeutic candidate for the treatment of lung cancer.

**Fig. 8:** Model of the GKB-induced anti-tumor effect in lung cancer cells. GKB acts as an anti-tumor agent that induces autophagy in lung tumor cells, which depends on beclin-1 and is associated with the inhibition of NLRP3-related inflammation

## Supplementary information

**Additional file 1 S-**Figure 1 *Ginkgolide B* (GKB) induced autophagy of lung cancer cells. Immunofluorescence analysis of the expression of the LC3B protein in lung cancer cells pretreated with CQ.

**Additional file 2 S-**Figure 2 *Ginkgolide B* (GKB) inhibited the proliferation, invasion and colony formation of lung cancer cells via beclin-1*.* The proliferation **(A)**, invasion (**B),** and colony formation **(C)** of Beclin-1-Si lung cancer cells treatment with GKB

The article "Ginkgolide B inhibits lung cancer cells promotion via beclin-1-dependent autophagy" was retracted in 2023. Reasons: duplicated images; overlap with earlier publications; unreliable data; concerns about the images.

## Data Availability

The datasets used and/or analyzed during the current study available from the corresponding author on reasonable request.
